The article "Multislice Spiral CT Image Analysis and Meta-Analysis of Inspiratory Muscle Training on Respiratory Muscle Function" was published in 2021. Journal: J Healthc Eng.

# Multislice Spiral CT Image Analysis and Meta-Analysis of Inspiratory Muscle Training on Respiratory Muscle Function

**DOI:** 10.1155/2021/1738205

**Published:** 2021-06-23

**Authors:** Lijuan An, Baiyan Li, Dan Ming, Weizhan Wang

**Affiliations:** People's Hospital of Hengshui, Clinical Medicine Major, Hebei, Hengshui 053000, China

## Abstract

Respiratory muscle function has a significant effect on stroke. Stroke is one of the most common cardiovascular and cerebrovascular diseases in the clinic and has a significant impact on the quality of life of patients. Hemiplegia, cerebral hemorrhage, and even death can occur, mainly in the elderly. In this paper, we meta-analyzed the effect of inspiratory muscle training on respiratory muscle function. In this article, we used a topic search method to search for relevant literature on respiratory muscle training and obtained 58 and 32 literature studies from CNKI and Wanfang Data, respectively. As a result of the screening, 36 and 28 documents were obtained. In this paper, 64 selected articles were studied. The authors make statistics on the literature of designing serum content index and multislice spiral CT (Member of the Society of Cardiological Technicians) image of patients, so as to analyze the influence of CT image and inspiratory muscle training on respiratory muscle function. The study showed that FVC, FEV1, MIP, and diaphragm mobility of the experimental group were significantly improved after treatment in more than 85% of the studies (*P* < 0.05), while those of the control group were not significantly improved (*P* > 0.05). The comparison between the two groups after treatment showed that FVC, FEV1, MIP, and diaphragm mobility of the experimental group were higher than those of the control group (*P* < 0.05). The application of multislice spiral CT image analysis technology can effectively evaluate the effect of inspiratory muscle training on respiratory dysfunction in stroke patients, the mechanism of which regulates the expression of related pathways, suppresses the inflammatory response, and can reduce oxidative stress damage. Therefore, respiratory muscle training can improve the function of respiratory muscle and reduce the death rate of cerebellar hemorrhage in patients with stroke and other vascular diseases.

## 1. Introduction

Stroke is one of the common cardiovascular and cerebrovascular diseases in clinic, which has a great impact on the quality of life of patients. It can easily cause hemiplegia, cerebral hemorrhage, and even death, mostly in the elderly. Stroke patients are prone to respiratory dysfunction, pulmonary infections, and other clinical symptoms, which show some resistance to the patient's treatment, primarily associated with diminished diaphragmatic function and activity. The diaphragm is an important respiratory muscle in the human body and accounts for 60% to 80% of the total respiratory muscle function. Stroke patients have neuronal damage and blockage of conduction pathways that affect diaphragm thickness and functional mobility.

The article "Multislice Spiral CT Image Analysis and Meta-Analysis of Inspiratory Muscle Training on Respiratory Muscle Function" was published in 2021. Journal: J Healthc Eng.

The onset of stroke is closely related to the inflammatory response. Atherosclerosis is the pathological mechanism of stroke. The development and progression of atherosclerosis is primarily associated with the inflammatory response. Schlattmann et al. pointed out that severe muscular respiratory muscle injury often requires glenoid muscle grafting to restore the area of respiratory muscle and maintain the stability of respiratory muscle [1]. Bradley proposed to treat severe muscular respiratory muscle surgery. At present, arthroscopic or open respiratory muscle surgery is commonly used in clinical practice, and iliac muscle block transplantation and tibial muscle allograft with articular surface are taken [2]. Sun et al. suggested that coracoid muscle block should be removed for transposition in respiratory muscle surgery. The coracoid process has multiple tendons and ligaments attached to it, which is an important part of maintaining the stability of the anterior superior part of the respiratory muscle. Intercepting the coracoid process for transposition destroys the normal anatomical structure of the coracoacromial arch in the coracoid process and affects the stability of the anterior superior part of the respiratory muscle [3]. According to Wang et al., the overall incidence rate of postoperative complications of respiratory muscle surgery is 6.1%∼30%, such as nerve injury, coronoid muscle fracture, muscular arthritis, and other surgical complications [4]. Teramoto et al. proposed that although the technique of iliac muscle graft is mature, it has two surgical sites, and the incidence of peripheral nerve injury is 5.8%, and the incidence of postoperative pain in donor site is 6.9% [5].

In the direction of training, Huang et al. proposed that the lower tibial muscle allograft has the advantages of certain radian and soft muscle surface, which can better restore the shape and function of the respiratory muscle pelvis. However, the preservation and transportation conditions of the lower tibial muscle allograft are strict, and the problems of immune rejection and potential disease transmission need to be further studied [6]. Zhang et al. proposed treating severe muscle respiratory muscle injury; the source of excellent muscle graft materials has become an important topic. However, the location of autologous respiratory muscle is shallow, far away from the neurovascular distribution area, and the normal anatomical structure of coracoid process is preserved, which has no obvious effect on the function and stability of respiratory muscle [7]. Vogel measured the length, width, and height parameters of respiratory muscle and coracoid process through CT three-dimensional reconstruction, which provided a reference for autologous respiratory muscle as the donor site of muscle mass [8]. Feng et al. suggested that the anterior and inferior respiratory muscle sacs of the respiratory muscle were loose and lack the blocking effect of muscle and muscle ilium, so the anterior dislocation of the respiratory muscle was the most common. The common cause of anterior respiratory muscle dislocation in young patients is respiratory muscle injury [9]. Gandolfi et al. proposed that multiple anterior dislocation of respiratory muscle further resulted in the destruction of respiratory muscle capsule and the defect of labrum muscle, resulting in muscular Bank Art injury [10]. The above research is from the medical clinical point of view of respiratory muscle training and injury recovery research, but the analysis of the training effect is lack of data; in addition, there is no combination of medical CT images for pathological speculation, so this paper is based on training, combined with CT images of respiratory muscle training for meta-analysis.

The article "Multislice Spiral CT Image Analysis and Meta-Analysis of Inspiratory Muscle Training on Respiratory Muscle Function" was published in 2021. Journal: J Healthc Eng.

In this paper, the effect of inspiratory muscle training on respiratory muscle function was meta-analyzed. In this paper, the topic search method was used to search the related literatures of respiratory muscle training, and 58 and 32 literatures were obtained from CNKI and Wanfang Data, respectively. As a result of the screening, 36 and 28 documents were obtained. In this article, 64 selected articles were studied. In this paper, the authors produced statistics on the patient's serum content index and literature for designing multislice spiral CT images and analyzed the effects of CT images and inspiratory muscle training on respiratory muscle function.

## 2. Meta-Analysis and CT Image Processing of Respiratory Muscle Training

### 2.1. Respiratory Muscle Training

Respiratory muscle pelvis with large muscular defect can be “inverted pear shape.” Based on the respiratory muscle CT, the optimal circle of the shoulder glenoid simulates the size of 25% of the muscular defect; that is, the width is 25% of the transverse diameter of the respiratory muscle glenoid. The shape of the respiratory muscles is fusiform. The initial part of the respiratory muscles is slender and becomes wide at the mid-spinal bulge (a wider protrusion on the inner side of the respiratory muscles about 4 cm). The respiratory muscles gradually widened from the spine bulge to 8 cm inside the respiratory muscles [11]. The position of the respiratory muscles is superficial, making it easier to take muscles. The suprascapular nerve and suprascapular artery are distributed on the outside and base of the respiratory muscles, while the 4∼8 cm area inside the respiratory muscles is located in the middle of the respiratory muscles, which is far from the neurovascular distribution area, which can avoid nerve and blood vessel damage during muscle removal. Respiratory muscle training describes the use of respiratory muscle training to treat the posterior glenoid instability, and the use of cadaver specimens to verify the biomechanics of respiratory muscle training to treat the posterior glenoid defect can reconstruct the stability of the posterior glenoid [12]. However, there are few reports in the literature on whether the respiratory muscles have sufficient muscle mass to meet the needs of severe muscle Bankart muscle grafts [13]. The first concept of using respiratory muscle training to treat respiratory muscle damage was proposed. Patients with bank cart muscle injury underwent autologous respiratory muscle harvesting and muscle transplantation and fixed their muscles using self-developed allogeneic cortical muscle crossing nails. Respiratory muscle injury has achieved satisfactory results, and the muscle grafts and the shoulder glenoid heal and remodel well [14]. The allogeneic cortical muscle has good tissue compatibility with the cross-nail, and its elastic modulus is also close to the skeletal tissue, which can eventually achieve crawling replacement [15].

The article "Multislice Spiral CT Image Analysis and Meta-Analysis of Inspiratory Muscle Training on Respiratory Muscle Function" was published in 2021. Journal: J Healthc Eng.

In this paper, through CT three-dimensional reconstruction, 120 scapular muscles were measured, which provides reliable data for autologous breathing muscles and muscle grafts. Through experimental data measurement, it is found that the average length of the respiratory muscle is about 12 cm, and the muscle area is 4 cm–8 cm inside the respiratory muscle, which is in the middle of the respiratory muscle [16]. The respiratory muscles gradually widen from the inside to the outside. The study found that male respiratory muscles are generally longer than female respiratory muscles, and the muscle mass is more sufficient [17]. Compared with the commonly used coracoid transposition in clinical practice, it is found that the respiratory muscles have sufficient muscle mass in terms of the length and height of the muscles [18]. Although the width of the respiratory muscle at the medial 4 cm is smaller than the coracoid process, it is significantly larger than the degree of the respiratory muscle defect, which has met the needs of muscle implantation for severe muscular respiratory muscle injury [19].

The article "Multislice Spiral CT Image Analysis and Meta-Analysis of Inspiratory Muscle Training on Respiratory Muscle Function" was published in 2021. Journal: J Healthc Eng.

### 2.2. Multislice Spiral CT Image Analysis Method

The electromagnetic wave CT detection method mainly uses the difference of electromagnetic wave absorption capacity of different media to predict the abnormal media in the propagation area according to the strength of the collected electromagnetic wave signal [20]. In the process of electromagnetic wave propagation in the same medium, the radiation intensity is mainly related to the transmission power and the combination form of antenna [21]. Therefore, when choosing the form of antenna, it is necessary to comprehensively consider the best matching form required for detection, so as to maximize the radiation energy [22]. In underground detection, due to the limitation of the working face construction conditions, the antenna with simple direction factor is usually considered, so the magnetic dipole antenna is selected to generate electromagnetic wave *e*:

(1) $$\begin{array}{c} E=\frac{\sum_{j=1}^{k}\sum_{h=1}^{k}\sum_{t=1}^{n_{j}}\sum_{r=1}^{n_{h}}\left|y_{ij}-y_{hr}\right|}{2n^{2}u}. \end{array}$$

When the electromagnetic wave radiation source propagates in isotropic and uniform medium, the electromagnetic wave field strength *e* at point *P* is

(2) $$\begin{array}{c} Ew=\sum_{j=1}^{k}G_{jj}p_{j}s_{j}, \end{array}$$

where *E* is the field strength measured at a distance *r* from the emission point in the propagation medium, microvolt (*µ* V); *E*0 is the initial field strength generated by electromagnetic wave transmitting end:

(3) $$\begin{array}{c} E_{t}=\overset{k}{\underset{j=2}{\sum }}\sum_{h=1}^{j-1}G_{jh}\left(p_{j}s_{h}+p_{h}s_{j}\right)D_{jh}\left(1-D_{jh}\right),\\ R_{jh}=\int_{0}^{\infty }\text{d}F_{h}\left(y\right)\int_{0}^{y}\left(y-x\right)\text{d}F_{j}\left(y\right),\\ E_{0}\left(x\right)=\frac{1}{Nh}\sum_{i=1}^{N}\left(\frac{X_{i}-x}{h}\right). \end{array}$$

Under the field space condition of electromagnetic wave CT detection in working face, *θ*, it can be approximated to 90. The formula for calculating the field strength *e* becomes

(4) $$\begin{array}{c} E\left(x\right)=\frac{1}{\sqrt{2\pi }}\theta \left(-\frac{x^{2}}{2}\right). \end{array}$$

When performing electromagnetic wave CT detection on a coal mine work surface, the electric field strength value collected by the receiver is always *h* (DB). Therefore, equation (4) is obtained in decibels.

(5) $$\begin{array}{c} H=\sigma t=\frac{\sqrt{\left(1/n\right)\sum_{i=1}^{n}{\left(FI_{it}-FI_{it}\right)}^{2}}}{FI_{it}},\\ B_{\left(j|i\right)}=w_{ij}X_{i},\\ H0_{j}=\sum_{i}c_{ij}u_{\left(j|i\right)}, \end{array}$$

where *H* is the field strength value recorded in the measurement, in db; *H*0 is the initial field intensity of emission, in dB. In the inversion calculation of electromagnetic wave tomography, firstly, the target detection area of coal mining face is discretized by grid, assuming that it is divided into *B* grids [23]. Each grid is called a pixel, and *XJ* is used to represent the real absorption coefficient of the *j*th grid [23]. Assuming that the total number of rays is a, then any ray passing through the detection area from the transmitting end to the receiving end will have an intercept of *D* on the *j*-th grid, and there will be

(6) $$\begin{array}{c} \ln\left(\frac{D_{it}}{D_{it}-1}\right)=\alpha +\beta \;\ln\;D_{it}-1+v_{i}+{ℑ}_{t}, \end{array}$$

where *Hi* is the electromagnetic wave field strength data collected by the *i*-th ray. The process of electromagnetic wave CT detection in working face is to emit electromagnetic waves at multiple emission points, so formula (6) can be further extended to

(7) $$\begin{array}{c} h_{t}=\tan h\left(w_{c}x_{t}+u_{c}\left(r_{t}\Theta h_{t-1}\right)+b_{c}\right). \end{array}$$

That is, it is the intercept of each ray passing through each grid, where the number of rays is a, and the number of grids is *B*. The unknown coefficient matrix of order *x*-*B∗*1 is the electromagnetic wave absorption coefficient of each pixel:

(8) $$\begin{array}{c} E_{j}=\frac{1/2u_{j}\sum_{i=1}^{n_{j}}\sum_{r=1}^{n_{j}}\left|y_{ji}-y_{jr}\right|}{n_{j}^{2}}, \end{array}$$

where *x* is the target value to be retrieved, that is, the absorption coefficient of each pixel. Due to the limitation of on-site detection conditions of coal mine working face, the number of rays is generally far less than the number of grids, so the solution of a sparse matrix with ill-conditioned characteristics is often needed [24]. There is no unique solution, and the current common art, sirt, and other traditional tomographic inversion algorithms mostly rely on the linearized form of the problem, using a single initial model; by repeatedly moving to the improved adjacent solution set, the inversion result largely depends on the selection of the initial value [25]. To solve this problem, this paper transforms the matrix solving problem into a functional extremum solving problem, establishes an objective function inversion model, and then solves the objective function through an intelligent algorithm with strong global search ability. In the process of electromagnetic tomography inversion, the objective function is often defined as the difference between the observed data and the theoretical data. Firstly, according to the formula, the measured loss value of field strength in the process of electromagnetic wave propagation is obtained. Then, a random initial absorption coefficient is given to the dielectric grid in the detection range, and the theoretical loss value of the field strength in the process of electromagnetic wave propagation is calculated. Finally, the absorption coefficient value of each grid is updated repeatedly by intelligent algorithm until the minimum objective function value or the number of iterations reaches the set upper limit; that is, the stop condition is satisfied, and the absorption coefficient value of each grid at the current time is output as the inversion result. The specific objective function is defined as follows:

(9) $$\begin{array}{c} I_{B}=\frac{\sum_{Z=1}^{h_{j}}\sum_{r=1}^{n_{h}}\left|y_{ji}-y_{hr}\right|}{n_{j}n_{h}\left(u_{j}+u_{h}\right)},\\ E_{nb}=\sum_{j=2}^{k}\sum_{h=1}^{j-1}G_{jh}\left(p_{j}s_{h}+p_{h}s_{j}\right)D_{jh}, \end{array}$$

which is the absorption coefficient vector to be inversed. Therefore, the tomographic inversion model of geological anomaly can make

(10) $$\begin{array}{c} h_{t}=z_{t}\Theta h_{t-1}+\left(1-z_{t}\right)\Theta h_{t}. \end{array}$$

When *HT* is the objective function and *f* (*x*) reaches the minimum value, *Z* and *H* corresponding to each grid are the upper and lower limits of variable variation. SGA is a global optimization random search intelligent algorithm, and its search performance mainly depends on the crossover operator and mutation operator with probability properties. Because SGA often adopts a single fixed genetic parameter, the selection of genetic parameters is particularly important. When using SGA to solve a variety of specific problems, scholars from different industries have proposed different ways to determine the values of genetic parameters, but so far, unified parameter selection rules have been adopted. That is, there is none. When faced with new optimization problems, you often need to do a lot of testing to choose the best results. However, not only is it time consuming, it is also not the best solution overall. Therefore, in order to avoid as early a convergence as possible when solving the objective function model of electromagnetic tomography inversion using the SGA intelligent algorithm, this paper guarantees SGA-based population diversity (global search performance). Therefore, in order to obtain a more accurate tomographic image inversion result, the search accuracy (local search performance) is improved as much as possible.

The article "Multislice Spiral CT Image Analysis and Meta-Analysis of Inspiratory Muscle Training on Respiratory Muscle Function" was published in 2021. Journal: J Healthc Eng.

## 3. Experimental Design

### 3.1. Research Methods

In this paper, the effect of inspiratory muscle training on respiratory muscle function was meta-analyzed. In this paper, the topic search method was used to search the related literatures of respiratory muscle training, and 58 and 32 literatures were obtained from CNKI and Wanfang Data, respectively. After screening, 36 and 28 literatures were obtained. In this paper, 64 selected articles were studied. The authors make statistics on the literature of designing serum content index and multislice spiral CT image of patients, so as to analyze the influence of CT image and inspiratory muscle training on respiratory muscle function.

### 3.2. Experimental Design

The CNKI search strategies of this meta-analysis are as follows:

  SU = respiratory muscle training
  TKA = “ct imaging diagnosis”
  AB% “functional training” and CF >20

For the selection of literature, although the length of the muscle was set as 4 cm, the length of 2-3 cm and the height of 1 cm can be selected according to the degree of muscle parenchyma defect. In this way, the attachment points and membrane of respiratory muscles need to be removed. It is necessary to repair the part of the respiratory muscle and suture the muscle. Because the intercepted muscle mass is small, and the attachment area of respiratory muscle is wide, it has little effect on muscle function. The body surface of the operation area can be marked along the respiratory muscle, and the respiratory muscle can be divided into three equal parts. About 3 cm incision was made from the middle part of the marked respiratory muscle. Prior to muscle transplantation, the shoulder pelvic defect should be refreshed with a spatula, and then the muscle block should be repaired to match the shape of the shoulder pelvis and the cortical muscles at the joints of the muscle block and shoulder pelvis should be repaired. Depending on the quality of the muscle and the shape of the defect, the direction of implantation should be adjusted, so that the muscle block fits into the defect in the respiratory muscle pelvis. This will help heal the injured area. Although the respiratory muscles have proven to have sufficient muscle mass, they can be used as a source of muscle transplantation for myogenic respiratory muscle injuries. However, some respiratory muscles have some morphological changes. To avoid side effects due to individual differences such as muscle weakness, muscle loosening, and lack of muscle mass, it is necessary to evaluate the muscle quality of the respiratory muscles before muscle transplantation.

There was no significant difference between the length of muscle and coracoid process (*P* > 0.05), and the length of respiratory muscle was (40 ± 4.5) mm, which was larger than the longitudinal diameter of glenoid (34.12 ± 3.79) mm. It is suggested that the length of the muscle to be taken from the respiratory muscle can meet the needs of the muscle graft in myogenic respiratory muscle injury. There was no significant difference between the width of the lateral part of the respiratory muscle and the width of the coracoid process. The width of the respiratory muscle was (9.76 ± 94) mm greater than 25% of the glenoid transverse diameter, which was the width of glenoid defect (6.44 ± 0.82 mm) (*P* < 0.001). The width of the lateral side of the respiratory muscle was (12.69 ± 84 mm) greater than 25% of the glenoid transverse diameter, which was the width of glenoid defect (6.44 ± 0.82) mm. It is suggested that the width of the muscle to be taken from the respiratory muscle can meet the needs of muscle grafting in muscular Bankart injury. The height of the medial side of the respiratory muscle was (17.67 ± 18) mm, higher than the height of coracoid process (9.40 3 ± 1.54) mm. The height of the lateral side of the respiratory muscle was (25.39 ± 86) mm, higher than the height of coracoid process (9.40 ± 1.54) mm. It is suggested that the height of muscle graft can meet the needs of muscle graft in patients with myogenic respiratory muscle injury. Respiratory muscle is the most flexible and unstable respiratory muscle in human body. 40% of the total respiratory muscle dislocation is respiratory muscle dislocation.

The article "Multislice Spiral CT Image Analysis and Meta-Analysis of Inspiratory Muscle Training on Respiratory Muscle Function" was published in 2021. Journal: J Healthc Eng.

## 4. Results and Discussion

### 4.1. Situation of Breathing Muscle Training in the Literature

As shown in Figure 1, delayed hemorrhage occurred in 4 patients within 3 months after operation, which were improved after renal artery interventional embolization. One patient had urinary fistula, which was improved after double-J tube implantation. Since the follow-up, 4 patients have recurred, and all of them have undergone secondary operation to remove the affected kidney and recurrent focus. One patient with multiple renal cell carcinoma underwent unilateral laparoscopic partial nephrectomy and oral sorafenib targeted therapy. The respiratory muscle status was stable.

As shown in Figure 2, the increasing number of patients with renal respiratory muscle injury poses great challenges to surgeons. BMI is not directly related to the difficulty of rlpn because it is an assessment of systemic fat and cannot accurately reflect the status of fat around the kidneys, another important factor in predicting the difficulty of surgery. Incidence of APF ranged from 10.6% to 40.8%, which was primarily associated with the systemic chronic inflammatory condition of metabolic syndrome.

As shown in Table 1, the AI assisted training system only provides preliminary training opinions for imaging physicians, and the final results will be reported by imaging physicians and bear corresponding responsibilities. But in the future, it is necessary to divide the responsibility scope of medical institutions, doctors, and AI enterprises from the legal level and define and investigate the responsibility in case of medical accidents.

The article "Multislice Spiral CT Image Analysis and Meta-Analysis of Inspiratory Muscle Training on Respiratory Muscle Function" was published in 2021. Journal: J Healthc Eng.

As shown in Table 2, the results show that the AI assisted training system based on CT image has high value in the training of respiratory muscle and can be used as a method of training respiratory muscle in clinical application. Integrating CT images, pathology, patients' past history, clinical characteristics, doctor training, patients' follow-up, and other data into AI assisted training system is the future development direction of AI. This will not only improve the accuracy of respiratory muscle training and reduce the workload of doctors, but also change the current medical mode, to promote the balanced development of medical resources in China.

As shown in Figure 3, the proportion of patients with hypertension and diabetes mellitus in map (mean arterial pressure) group increased significantly, accounting for 42.9% (66/154) and 56.5% (87/154), respectively, which may be related to systemic inflammatory reaction, chronic exudation of blood vessels around hypertension or diabetic small vessel disease. The thickness and density of APF can be accurately measured by preoperative CT and can be quantified according to map score. Although robotic laparoscopic surgery has obvious advantages, high map score in laparoscopic partial nephrectomy can significantly increase the time of fat separation. No previous study compared the difficulty of map score and intraoperative fat separation time in predicting rlpn.

As shown in Figure 4, the fat separation time and operation time of high map group were significantly higher than those of medium map group and low map group, indicating that high preoperative map score can predict the difficulty of rlpn operation. The higher the map score, the more estimated the blood loss. It was also found that the operation time of high map group was longer than that of low map group, and the intraoperative blood loss was more. The main reason was that the time of separating the renal pedicle, freeing the kidney and exposing the fat around the respiratory muscle, was significantly longer, and the blood vessels in the fat were bleeding during the separation and cutting process, which increased the estimated blood loss.

As shown in Figure 5, in addition to the map score alone, the combined score or the new scoring system seems to be more predictive. Map score is an important predictor of intraoperative blood loss, operation time, and intraoperative complications in rlpn, and its combined renal score is better than single score in predicting intraoperative complications. However, we found that there was no significant increase in postoperative complications in high map group, which may be related to the rich experience of rlpn.

The article "Multislice Spiral CT Image Analysis and Meta-Analysis of Inspiratory Muscle Training on Respiratory Muscle Function" was published in 2021. Journal: J Healthc Eng.

As shown in Table 3, map score is significantly correlated with CT thickness of posterolateral and medial perirenal fat and diabetes mellitus. It is considered that this radiologic clinical scoring system has better predictive value than map score alone. RNP score combined with the advantages of renal score and map score has good predictive value for rlpn operation time, estimated blood loss, positive margin, ischemic time, and complications, and the consistency between observers is good.

As shown in Figure 6, before tomographic inversion of the electromagnetic wave CT data collected by the working face, the detection area of the working face is discretized by grid. In order to ensure that each ray can be distributed inside the grid, the size of each grid is defined as 10.3 M × 3 m, 470 grids in total. On the basis of prior data of two lanes and borehole exposure in working face, based on average value constraint and CT recognition intelligent algorithm, after 500 generations of search evolution, the objective function value finally converges to 2.605 dB/m, as shown in Table 4.

Because the foreground background ratio is unbalanced, as shown in Table 4, Region of Interest (ROI) extraction can also be used to maintain the ratio of positive and negative samples when intercepting patches. The model can better learn the CT image features, images with unbalanced categories. For example, some doctors focus on the whole, while others focus on the details. To adapt to the different needs of film reading, this paper uses an improved network based on 3D U-net as the muscle frame network and inputs intercepted voxel patches into high and low resolution muscle frame networks. It is for training (the two receptor areas are different) and learns the overall and detailed features of lung CT images. The following is a detailed description of the segmentation network.

As shown in Figure 7, the segmentation network is divided into three parts: preprocessing module, muscle frame network, and integrated learning. In the preprocessing part, the original CT image is resampled in the *z*-axis, and then the data is amplified. Because the data layer thickness is not sparse, and the feature difference is obvious, this paper takes three-dimensional voxel patch for the amplified data set, so that the network can share parameters in three dimensions, so as to learn the difference of each dimension more accurately. At the same time, because the size of the input image in the three dimensions may be different, we need to use a fixed size voxel patch to make the model compatible with different sizes of input images on the plane.

The article "Multislice Spiral CT Image Analysis and Meta-Analysis of Inspiratory Muscle Training on Respiratory Muscle Function" was published in 2021. Journal: J Healthc Eng.

As shown in Figure 8, the data amplification methods used in this paper include scaling rotation, brightness enhancement, gaussian noise, and gamma correction, which are commonly used in natural image processing, as well as mirror flipping, which is commonly used in medical images. Considering that the size of lesions in multisite CT images is variable and uneven, which brings difficulties to network learning, the data amplification method in this paper does not use elastic transformation and other data amplification methods to avoid data leakage. Finally, in the preprocessing stage, we extract ROI from the amplified data to alleviate the problem of category imbalance; that is, when extracting 3D voxel patches, we intercept the foreground focus area with a certain proportion, so that the number of randomly cropped foreground background voxels is balanced.

The improved model based on 3D u-net is shown in Tables 5 and 6. Two muscle frame networks of the same system, low resolution network and high resolution network, are adopted, respectively. Compared with high-resolution network, low-resolution network has fewer codec layers and lower semantic level of segmentation. Batch normalization normalizes the data of each batch to a normal distribution with learnable parameters, which can reduce the deviation of data distribution and accelerate the convergence of neural network. Compared with the case normalization method, the batch normalization method removes the batch and channel and calculates the learnable parameters for each channel of each sample separately. Although it increases the cost of calculation, it can effectively improve the segmentation effect and maintain the independence between different samples in the same batch and different channels in the feature map. Based on this, this paper uses example normalization in the network.

As shown in Figure 9, in more than 85% of the studies, FVC, FEV1, MIP, and diaphragmatic mobility of the experimental group after treatment were significantly higher than those before treatment (*P* < 0.05), while the above indexes of the control group were not significantly improved (*P* > 0.05). The comparison between the two groups after treatment showed that FVC, FEV1, MIP, and diaphragmatic mobility of the experimental group were higher than those of the control group (*P* < 0.05). The application of multislice spiral CT image analysis technology can effectively evaluate the effect of inspiratory muscle training on respiratory dysfunction in stroke patients, and its mechanism can regulate the expression of related pathways, inhibit inflammatory response, and reduce oxidative stress injury. Therefore, respiratory muscle training can improve the function of respiratory muscle and reduce the death rate of cerebellar hemorrhage in patients with stroke and other vascular diseases.

The article "Multislice Spiral CT Image Analysis and Meta-Analysis of Inspiratory Muscle Training on Respiratory Muscle Function" was published in 2021. Journal: J Healthc Eng.

### 4.2. Discussion

Stroke is a common cardiovascular and cerebrovascular disease, and its neurological function is impaired. The incidence rate of the global is higher. The etiology may be related to hypertension and hyperlipidemia. The pathogenesis is complex, the cure rate is low, and the complications can easily cause death. Long time mechanical ventilation can easily cause diaphragm dysfunction. Diaphragmatic dysfunction may be related to primary lesion damage, respiratory center damage, secondary injury caused by complications, iatrogenic injury caused by mechanical ventilation, etc. Studies have shown that inspiratory muscle training can effectively improve the diaphragm function, which is widely used in clinical practice. Respiratory muscle strength is an important indicator of lung function in vivo, which can improve the function of stroke patients through inspiratory muscle training. The maximum strength of inspiratory muscle represents MIP, which can reflect the strength degree of inspiratory muscle. The movement degree of diaphragm reflects the damage degree of diaphragm function, which can significantly reflect the lung function of stroke patients. The changes of hs CRP content in patients with stroke are positively correlated with the degree of brain tissue damage, which can predict whether patients lead to death or disability. IL-6 can also be used as a marker of severity in stroke patients and as one of the injuries. IL-6 regulates the expression of related inflammatory factors such as TNF-H. CRP can further accelerate the development of inflammatory reactions. In addition, TNF-*α* expression reflects the degree of lung infection and is an independent risk factor for other complications. At the onset of stroke, brain tissue is damaged, and cells release reactive oxygen species (ROS) and inflammatory factors to cause an inflammatory reaction, which in turn causes nerve cell apoptosis and inhibits the functioning of nerve functions. The expression of SOD and GSH PX reflects the ability of the human body to remove ROS.

## 5. Conclusions

Multislice spiral CT is widely used in the evaluation of airway anatomy because of its high spatial resolution and nearly isotropy. Through multiplanar reconstruction of airway CT image and adjusting the tilt angle, any section of airway can be obtained, so it is helpful to measure airway from all angles. In previous studies, the measurement of laryngeal airway was mostly based on CT cross-sectional images of larynx. However, because the cross section of the laryngeal airway is not perpendicular to the median line of the larynx, the measurement of the airway diameter through the cross section is not accurate. In this paper, multiplanar reconstruction of neck CT was performed. After adjusting the tilt angle, the views of respiratory muscle and annular soft muscle strictly perpendicular to the median line of larynx were obtained. Therefore, the inner diameter of airway can be accurately measured. However, the results also show that the inferior diameter of respiratory muscle is less than the transverse diameter of annular soft muscle, which means that the larynx is inverted funnel-shaped on the coronal plane. It was also found that there was no correlation between the ratio of the inner diameter of the lower respiratory muscle to the inner diameter of the annular soft muscle and age, which indicated that there was no significant change in the morphology of the larynx during growth and development. It is found that the transverse diameter of the lower respiratory muscle is the narrowest part of the larynx. However, up to now, most of the studies on the type of tracheal intubation in children are based on the transverse diameter of the cricoid soft muscle. The lower part of respiratory muscle is composed of soft tissue with good compliance. The cricoid muscle is the only closed soft muscle ring in the airways and is poorly compliant, so the cricoid muscle is the narrowest part of the function and determines whether it can pass through the larynx. In this paper, combining software measurement data with sample measurements further enhances the content of the study. In the future, we will improve related research by combining sample measurement data and biomechanics. In conclusion, the length, width, and height of the autologous respiratory muscle graft can meet the needs of severe respiratory muscle injury. It can be used as a source of muscle transplantation for shoulder glenoid defects, providing a new option for clinical treatment of muscle respiratory muscle injury.

The article "Multislice Spiral CT Image Analysis and Meta-Analysis of Inspiratory Muscle Training on Respiratory Muscle Function" was published in 2021. Journal: J Healthc Eng.

## Figures and Tables

**Figure 1:** Respiratory muscle state after treatment.

**Figure 2:** The difficulty of BMI and RLPN.

**Figure 3:** Proportion of patients with hypertension and diabetes in the high group.

**Figure 4:** Fat separation time and operation time.

**Figure 5:** Joint scoring or new scoring system.

**Figure 6:** Electromagnetic wave CT data collected on the working face.

**Figure 7:** Segmentation network and preprocessing module.

**Figure 8:** CT multislice spiral image with natural image processing (some images are from the Internet and have been authorized by the authors to be available).

**Figure 9:** Inspiratory muscle training improves respiratory dysfunction in stroke patients.

**Table 1:** AI assisted training system.

Item	Expose	RLPN	Chronic exudation	Embolism	Respiratory muscles
Kidney part	3.41	2.84	3.76	3.58	2.23
Bleeding volume	2.78	5.34	3.46	4.18	3.51
AI assisted	2.6	4.85	3.23	3.98	4.96
Renal pedicle	2.27	1.61	1.51	2.28	1.97
Free kidney	4.62	3.2	4.93	6.3	6.38
Diabetes	6.66	2.55	6.45	1.76	5.47

**Table 2:** The role of AI-assisted training system in the training of respiratory muscles.

Item	RNP	MAP	3D U-net	Laparoscopy	Kidney part
Diabetes	2.76	2.92	3.03	2.67	3.11
Expose the tumor	2.85	4.68	2.41	4.13	5.17
RLPN	2.38	2.95	3.28	4.51	4.89
Chronic exudation	4.56	4.01	5.28	3.32	6.72
Kidneys	4.38	1.83	5.26	4.5	1.63
Respiratory muscles	5.2	4.74	3.77	6.79	2.44

**Table 3:** MAP score and posterolateral.

Item	CT recognition	Search evolution	RNP	MAP	3D U-net
Bleeding volume	1.76	1.92	0.02	0.79	1.45
Fat	2.31	2.01	1.83	1.66	2.3
Renal pedicle	5.62	4.29	4.76	5.01	4.59
Free kidney	5.45	4.9	2.09	4.6	5.18
Diabetes	3.95	4.69	2.44	3.45	1.03
Upgrade	4.3	1.55	5.04	1.44	1.64

**Table 4:** The objective function value finally converges.

Item	Expose the tumor	RLPN	Chronic exudation	Embolism	Kidneys
Bleeding volume	4.27	5.96	4.46	5.16	4.29
Fat	5.57	5.8	4.57	3.22	5.43
Renal pedicle	3.75	3.06	1.95	3.95	2.21
Free kidney	4.64	4.99	5.68	5.1	6.73
Diabetes	6.07	5.79	5.65	2.47	2.96

**Table 5:** Improved model of 3D U-net.

Item	CT recognition	Search evolution	RNP	MAP	3D U-net
Laparoscopy	1.48	1.95	3.8	3.64	2.05
Kidney part	4.96	5.08	3.16	4.66	3.36
Bleeding volume	3.86	5.04	2.25	2.28	5.85
Fat	3.27	4.14	2.3	1.5	2.32
Renal pedicle	1.51	2.78	3.06	4.16	5.73
Free kidney	6.8	1.6	6.32	2.33	5.66

**Table 6:** Low-resolution network and high-resolution network.

Item	Laparoscopy	Kidney part	Bleeding volume	Fat	Renal pedicle
Diabetes	0.63	0.15	1.27	1.38	0.97
Expose the tumor	3.82	1.51	2.54	3.06	1.64
RLPN	4.94	5.04	2.37	5.34	5.32
Chronic exudation	2.37	2.09	3.66	2.53	5.2
Embolism	1.27	3.07	1.29	1.08	1.21

## Data Availability

Data cannot be shared without permission from the data provider.
